RETRACTED

# Mitochondrial tRNA Mutations Associated With Essential Hypertension: From Molecular Genetics to Function

**DOI:** 10.3389/fcell.2020.634137

**Published:** 2021-01-22

**Authors:** Yuqi Liu, Yundai Chen

**Affiliations:** ^1^Cardiac Department, Chinese PLA General Hospital, Medical School of Chinese PLA, Beijing, China; ^2^Department of Cardiology & National Clinical Research Center of Geriatrics Disease, Chinese PLA General Hospital, Beijing, China; ^3^Beijing Key Laboratory of Chronic Heart Failure Precision Medicine, Chinese PLA General Hospital, Beijing, China; ^4^National Key Laboratory of Kidney Diseases, Chinese PLA General Hospital, Beijing, China; ^5^Cardiac Department, Chinese PLA General Hospital, Beijing, China

**Keywords:** tRNA, mtDNA, hypertension, maternal, mutation

## Abstract

Essential hypertension (EH) is one of the most common cardiovascular diseases worldwide, entailing a high level of morbidity. EH is a multifactorial disease influenced by both genetic and environmental factors, including mitochondrial DNA (mtDNA) genotype. Previous studies identified mtDNA mutations that are associated with maternally inherited hypertension, including tRNA^Ile^ m.4263A>G, m.4291T>C, m.4295A>G, tRNA^Met^ m.4435A>G, tRNA^Ala^ m.5655A>G, and tRNA^Met^/tRNA^Gln^ m.4401A>G, et al. These mtDNA mutations alter tRNA structure, thereby leading to metabolic disorders. Metabolic defects associated with mitochondrial tRNAs affect protein synthesis, cause oxidative phosphorylation defects, reduced ATP synthesis, and increase production of reactive oxygen species. In this review we discuss known mutations of tRNA genes encoded by mtDNA and the potential mechanisms by which these mutations may contribute to hypertension.

## Introduction

According to the 2018 European Society of Cardiology/European Society of Hypertension (ESC/ESH) Guidelines for the Management of Arterial Hypertension, the incidence of hypertension remains high (Williams et al., 2018). Although studies have shown that drug therapy and lifestyle changes can significantly lower blood pressure, hypertension is still poorly controlled worldwide, including in Europe, and remains the leading cause of cardiovascular disease (CVD) and all-cause death (Falaschetti et al., 2014). If the definition of hypertension were revised to a blood pressure (BP) of ≥130/80 mmHg, as suggested by the 2017 American College of Cardiology/American Heart Association (ACC/AHA) guidelines (instead of the JNC 7 definition, which is currently in use), the crude prevalence of hypertension in the United States would increase from 32% to 46% (from JNC7 guidelines to the 2017 ACC/AHA guideline Muntner et al., 2018). Applying these new diagnostic criteria for hypertension would also mean that, the prevalence of hypertension would be greater than 50% worldwide (Lu et al., 2017). Therefore, hypertension prevention and treatment represent a tremendous burden to the healthcare system.

RETRACTED

EH is a multifactorial disease that is influenced by both genetic and environmental factors, including the autonomic nervous system, vasopressor/vasodepresser homones, the structure of the cardiovascular system, body fluid volume, renal function and many others (Maolian and Norbert, 2006). Immune cell functioning and their interactions with tissues that regulate hypertensive responses may also contribute to hypertension (Justine et al., 2017; Rong et al., 2021). The role of genetic factors in its etiology was demonstrated by a cross-sectional analysis that showed familial aggregation despite environmental factors (Rice et al., 1989). The rate of genetic variance associated with EH has been estimated to range from 20% to 50% (Longini et al., 1984; Hunt et al., 1989) and both maternal (Friedman et al., 1988; Chung et al., 1999; DeStefano et al., 2001) and paternal patterns of inheritance (Hurwich et al., 1982; Rebbeck et al., 1996; Uehara et al., 1998) have been reported. Correlations between BP in mothers and their offspring, as well as maternally inherited hypertension, have been reported in several studies (Borhani et al., 1969; Bengtsson et al., 1979; DeStefano et al., 2001).

Fuents et al. found that there was a significant correlation between maternal hypertension and hypertension in progeny, and observed that some diseases caused by mtDNA mutation were accompanied by hypertension (Fuentes et al., 2000). Austin et al. studied a family with mitochondrial encephalomyophthy, lactic acidosis and stroke-like episodes syndrome (MELAS) and found that, in addition to clinical symptoms such as myoclonic and tonic myoclonic epilepsy, these patients often also had hypertension, suggesting that hypertension may be related to mtDNA mutations (Austin et al., 1998). Watson et al. also found that the incidence of the m. 10398A>G mutation in the mitochondrial ND3 gene and the m.6620T>C/m. 6260G>A (OMIM516030) double point mutation in the HaeIII CO1 gene was significantly higher in patients with hypertension-associated end-stage renal disease than in the control group (Watson et al., 2001). Liu et al. compared and analyzed gene changes in the D-loop region that regulates hypertension and normal blood pressure and found that the frequency of variation in the hypertension group was higher than that seen in the normal blood pressure group (Liu et al., 2005). These studies suggest that essential hypertension with maternal genetic characteristics may be related to mtDNA mutations.

RETRACTED

## Characteristics of the Mitochondrial Genome

The mammalian mitochondrial genome is a closed, circular, double-stranded, 16,569-bp molecule. The outer and inner rings comprise a G-rich heavy strand, and a C-rich light strand, respectively. The mitochondrial genome includes both coding and non-coding regions (D-loop). The coding region includes 37 genes that encode, 13 peptides associated with the oxidative phosphorylation (OXPHOS) respiratory chain complex, as well as 22 tRNAs and 2 rRNAs (12S rRNA and 16S rRNA) that are required for mitochondrial protein synthesis (Anderson et al., 1981). While mtDNA can be replicated, transcribed, and translated independent of the nucleus genome, mitochondrial function also relies on proteins encoded by nuclear DNA, including some structural proteins and some proteins involved in OXPHOS.

Only the mother's mitochondria are passed to the next generation, because sperm-derived mitochondria are targeted for selective destruction via mitophage-mediated ubiquitination shortly after oocyte fertilization (Al Rawi et al., 2011). Therefore, mtDNA is inherited from the mother, not the father, and mitochondrial-inherited diseases are always associated with the maternal lineage. Thus, the hereditary model for mitochondrial disease is not Mendelian, but rather is more analogous to the polygenic disease model, in which the degree of illness is associated with the extent of mitochondrial involvement.

MtDNA has no histones, and the repair system is imperfect, so mtDNA has a high rate of mutations induced by reactive oxygen species (ROS) produced during electron transport. In addition, every cell contains more than one mitochondrion, and each mitochondrion contains ~10–100 copies of the mitochondrial genome. Therefore, mtDNA heterogeneity is mutant and wild-type mtDNA which exist in a single cell at the same time, rather than all the mtDNA in the cell being homogeneous. Mitochondria with and without mutation separate rapidly during cell division, and ultimately mutant mtDNA found in each individual cell is homogeneous (Jenuth et al., 1996). The phenotype mainly depends on the ratio of mutant to wild-type mtDNA. The minimum number of copies of the mutant mtDNA that can cause specific tissue and organ dysfunction is called the threshold, and the phenotype is referred to as the mitochondrial threshold effect (Lu et al., 2017). If less than 60% of the mtDNA is mutated, then the phenotype is likely to be normal. However, if a greater proportion of the mtDNA is mutated, clinical symptoms, in some cases affecting multiple organs, can occur. The clinical phenotype is closely related to the severity of oxidative phosphorylation defects and the energy needs of individual organs. Different tissues and organs have varying numbers of mitochondria and percentages of mutant mtDNA. The frequency of mtDNA mutation is typically higher in the brain, skeletal muscle, heart, kidney, and liver compared with in the blood.

RETRACTED

Mitochondrial gene mutations include point mutations, deletions, insertions, and nuclear gene–mediated mutations (Yan and Guan, 2008), as well as copy number mutations. MtDNA mutation mainly affects mitochondrial energy production, leading to decreased synthesis of ATP and increased synthesis of ROS, and thus to a variety of mitochondrial diseases, such as deafness, neuropathy, myopathy, cardiomyopathy, diabetes, Alzheimer's disease, and Parkinson's disease (Schon et al., 1997; Wallace, 1999). Heterogeneous mtDNA mutations are more common in children, and tend to be associated with more severe clinical symptoms, such as mitochondrial myopathy. Homogenous mtDNA mutations can be found in patients with mild clinical symptoms and are often associated with common late-onset diseases (Wallace, 2000), such as Alzheimer's disease (Hutchin and Cortopassi, 1995), Parkinson's disease (Mayr-Wohlfarth et al., 1997), and type 2 diabetes (Perucca–Lostanlen et al., 2000). The phenotype associated with a mtDNA mutation is affected by various factors, such as nuclear genes (Li et al., 2002), mitochondrial haplotype (Brown et al., 2002), and environment (Prezant et al., 1993), and mitochondrial diseases therefore have variable presentations. Given that mtDNA mutations have the distinctive characteristics described above, and that hypertension is a common major disease caused by the interaction of multiple genetic and environmental factors, it is important to study the potential role of mitochondria in hypertension.

## The Mitochondrial Genome and Cardiovascular Disease

Although genes encoding mitochondrial tRNAs account for only 10% of the mtDNA, 320 amino acid changes associated with diseases have been identified that are caused by 831 mutations in mtDNA sequences encoding mitochondrial tRNAs (MITOMAP: A Human Mitochondrial GenomeDatabase 2020, http://www.mitomap.org).

In 2000, Andreu et al. (2000) first identified a G to A point mutation, which was associated with a Gly to Asp substitution, at residue 15498 (OMIM516020) of the mitochondrial gene encoding cytochrome b (MTCYB) in a patient with histiocytoid cardiomyopathy. Later, Schuelke et al. reported a patient with severe neurological symptoms and hypertrophic cardiomyopathy associated with a highly conserved mutation from T to C at residue 14849 (OMIM516020) of the MTCYB gene (Schuelke et al., 2002). In 2008, Jonckheere et al. reported a novel mutation (m.8529 G>A, OMIM516070) in the mitochondrial gene ATP8 that was associated with apical hypertrophic cardiomyopathy and neuropathy (Jonckheere et al., 2008). More recently, Ware et al. reported a family with hypertrophic cardiomyopathy and congestive heart failure associated with a T to C mutation at residue 8528 (OMIM516070), resulting in a Met to Thr substitution and Trp55 to Arg (Ware et al., 2009).

RETRACTED

Since Tanaka et al. (1990) first reported a case of fatal infant cardiomyopathy in a patient carrying a tRNA^Ile^ m.4317 A>G mutation (OMIM590045), multiple tRNA^Ile^ mutations associated with hypertrophic cardiomyopathy have been identified, including m.4269A>G (Taniike et al., 1992) (OMIM590045), tRNA^Leu(UUR)^ m.3303C>T (Silvestri et al., 1994) (OMIM590050), m.3260A>G (Mariotti et al., 1994) (OMIM590050), tRNA^Gly^ m.9997T>C (Merante et al., 1994) (OMIM590035), tRNA^Lys^ m.8363G>A (Santorelli et al., 1996) (OMIM590060), m. 4295A>G (Merante et al., 1994) (OMIM590045), tRNA^His^ m.12192G>A (Shin et al., 2000) (OMIM590040), m.4284G>A (45) (Corona et al., 2002) (OMIM590045) and m.4300 A>G (46) (Taylor et al., 2003) (OMIM590045). In addition to mutations in mitochondrial genes encoding tRNAs, a m.1555A>G mutation in the mitochondrial gene encoding 12S rRNA (OMIM561000) has also been reported in a woman with restrictive cardiomyopathy (Santorelli et al., 1999). Thus, altogether, one mutation has been identified in mtDNA encoding a small rRNA, which account for 6.25% of the mitochondrial genome; 11 mutations in sequences encoding tRNAs, which account for 68.75% of the mitochondrial genome; and four mutations in other protein coding regions accounting for 25% of the mitochondrial genome, suggesting that mitochondrial encoded tRNA genes are a cardiovascular disease-related mutation hotspot.

## The Molecular Genetics of mtDNA Mutations in EH

The Framingham Heart Study (FHS) reported that ~35.2% of hypertensive pedigrees are potentially associated with mitochondrial effects (Yang et al., 2007). This study showed a maternal effect on hypertension and quantitative systolic BP, providing further evidence for the influence of mitochondria on hypertension.

MtDNA encodes 22 tRNAs, including tRNA^Leu(UUR)^, tRNA^Gln^, tRNA^Ile^, and tRNA^Met^, and others. Eukaryotic tRNAs, which are predominantly nuclear-encoded, are 73–90 nucleotides (nt) long and have a clover leaf-shaped secondary structure. In human mitochondria, each tRNA corresponds to a single amino acid, with the exception of tRNA^Leu^ and tRNA^Ser^ (Suzuki et al., 2011). In addition, the secondary structure of mitochondrial tRNAs contains a significant amount of unstable nucleotide pairs, such as non–Watson-Crick pairs and A-U pairs. Taken together, these features mean that mitochondrial tRNAs have lower thermal stability and are more susceptible to mutation than nuclear-encoded tRNAs.

RETRACTED

Usually, the acceptor stem is 7 bp long, the anticodon (AC)-stem is 5 bp, and the D-stem is 3–4 bp. Although some tRNA species have a 4–12 nt D-loop and the variable (V) region, starting at residue 44, may be 4–23 nt long, the AC-triplet always starts from position 34–36 and the CCA tail always starts from position 74–76 (Figure 1A). These two regions are fundamentally important for delivering amino acids to the ribosome, then translating the genetic information in an mRNA template-directed manner into a corresponding polypeptide chain (Kirchner and Ignatova, 2015). Mitochondrial tRNA precursors are processed into mature tRNAs by a series of enzymes: RNase P processes the 5′ end, tRNase Z processes the 3′ end, CCAse adds the CCA tail to the 3′ end after 3′ endonuclease catalysis, then aminoacyl-tRNA synthetase (aaRS) adds amino acids to the end of the CCA tail, before final conversion into the mature mitochondrial tRNA (Figure 1) (Levinger et al., 2004).

**Figure 1:** Clover leaf-shaped secondary tRNA structure. **(A)** clover leaf-shaped structure includes the acceptor stem, D-loop, D-stem, anticodon (AC)-stem, AC-loop, T-loop, T-stem and variable (V) region. **(B–L)** tRNAs mutations associated with cardiac disease and EH.

### The tRNA^Ile^ m.4291T>C and m.4295A>G Mutations Are Associated With EH

The mitochondrial tRNA^Ile^ m.4291T>C (OMIM590045) mutation (Wilson et al., 2004) affects position 33 of tRNA^Ile^, adjacent to the 3′ end of the anticodon, which is highly conserved (Figure 2, Table 1). The U residue in the 33rd position of tRNA^Ile^ can form a hydrogen bond with the third base of the anti-codon (Quigley and Rich, 1976), forming an anti-codon loop, making the anti-codon easier to identify when bound to the homologous mRNA codon on the ribosome (Kim et al., 1973). When the mitochondrial tRNA^Ile^ m.4291T>C mutation is present, and the hydrogen bond between the 33rd position of tRNA^Ile^ and the 3rd position of the anticodon is destroyed, resulting in a failure of the formation the anti-codon loop, ultimately affecting the identification of the codon. The mitochondrial mutation tRNA^Ile^ m.4295A>C (OMIM590045) (Li et al., 2008) is located at residue 37th, adjacent to the 5′ end of the anticodon, which is highly conserved (Figure 1). This residue plays a very important role in anti-codon recognition and maintenance of the structure and the stability of tRNA^Ile^ (Björk, 1995).

RETRACTED

**Figure 2:** Post-transcriptional processing of a typical intron containing tRNA transcript. RNase P processes the 5′ end, tRNase Z processes the 3′ end, CCAse adds the CCA tail to the 3′ end after 3′ endonuclease catalysis, and aaRS adds amino acids to the end of CCA, thereby generating the mature mitochondrial tRNA (Levinger et al., 2004).

**Table 1:** MtDNA mutation associated with EH.

**Gene**	**Mutation**	**Disease**	**Aberrant mtDNA biology**	**OMIM**	**References**
12s RNA	m.1555A>G	Restrictive cardiomyopathy	Alteration of mitochondrial protein synthesis	561000	Santorelli et al., 1999
MT-TL1	m.3243A>G	Early ARM, mild hearing loss, hypertension, ischemic heart disease, and asthma	Unclear	590050	Jones et al., 2004
	m.3253T>C	Hypertension	Decreased in the steady-state level of tRNA^Leu(UUR)^	590050	Zhou et al., 2017
	m.3260A>G	Maternally inherited myopathy and cardiomyopathy	mtDNA-related respiratory capacity, including oxygen consumption, complex I- and complex IV-specific activities, and lactate production, were markedly abnormal.	590050	Mariotti et al., 1994
	m.3303C>T	Fatal infantile cardiomyopathy	Disrupts a conserved base pair in the aminoacyl stem of the tRNA^Leu(UUR)^	590050	Silvestri et al., 1994
MT-ND1	m.3308T>C	Adjacent sequence of MT-ND1 and tRNA^Leu(UUR)^	Alteration on the processing of the H-strand polycistronic RNA precursors; the destabilization of MT-ND1 mRNA; substitution p.Met01Thr.	516000	Liu et al., 2008
MT-TI	m.4263A>G	Maternally inherited hypertension	Reduction in the steady-state level of tRNA^Ile^; Decrease in the Level of Mitochondrial tRNA^Ile^; Mitochondrial Protein Synthesis Defect; ROS Production Increases	590045	Wang et al., 2011
	m.4269A>G	Dilated cardiomyopathy	Ragged red fibers and focal cytochrome C oxidase-deficient fibers in skeletal and cardiac muscles	590045	Taniike et al., 1992
	m.4284G>A	Cardiomyopathy	Lower complex I and IV activities		Corona et al., 2002
	m.4291T>C	Hypertension, hypercholesterolemia, and hypomagnesemia	Adjacent to the anticodon of tRNA^Ile^; a failure of the formation the anti-codon loop	590045	Wilson et al., 2004
	m.4295A>G	Maternally inherited hypertension	37 adjacent to the anticodon of tRNA^Ile^; Anticodon dysrecognition	590045	Li et al., 2008
	m.4295A>G	Hypertrophic cardiomyopathy	Respiratory chain dysfunction		Merante et al., 1994
	m.4300A>G	Hypertrophic cardiomyopathy	Low steady-state levels of the mature mitochondrial tRNA^Ile^	590045	Taylor et al., 2003
	m.4317A>G	Fatal infant cardiomyopathy	Defects of complex I and complex IV of the respiratory chain	590045	Tanaka et al., 1990
MT-NC2	m.4401A>G	Maternally inherited hypertension	Junction of tRNA^Gln^ and tRNA^Met^; RNase P reaction efficiency in tRNA^Met^ and tRNA^Gln^ 5′-end metabolism	590065	Li et al., 2009
MT-TM	m.4435A>G	Maternally inherited hypertension	Adjacent to the anticodon of tRNA^Met^; Reduction in the levels of tRNA^Met^; mitochondrial Protein Synthesis Defect	590065	Liu et al., 2009
tRNA^Ala^	m.5655A>G	Hypertension	Reduction in the steady-state level of tRNA^Ala^	590000	Jiang et al., 2016
MT-CO1	m.5913G>A	Hypertension	on average, 7-mm Hg higher systolic BP at baseline; amino acid change D5N in CO1	516030	Liu et al., 2012
	m. 6260G>A	Hypertension	Hypertension-associated end-stage renal disease	516030	Watson et al., 2001
	m. 6620T>C	Hypertension	Hypertension-associated end-stage renal disease	516030	Watson et al., 2001
tRNA^Asp^	m.7551A>G	Hypertension	Potential structural and functional alterations	590015	Xue et al., 2016
MT-TK	m.8363G>A	Hypertrophic cardiomyopathy	Defects of complexes I, III, and IV of the electron-transport chain.	590060	Santorelli et al., 1996
ATP8	m.8528T>C	Hypertrophic cardiomyopathy and congestive heart failure	p.Met01Thr in ATP8 and p.Trp55 Arg in ATP6	516070	Ware et al., 2009
	m.8529G>A	Apical hypertrophic cardiomyopathy and neuropathy	An improper assembly and reduced activity of the complex V holoenzyme; amino acid change of p.Trp55Arg in ATP6 and p.Met00Thr in ATP8	516070	Jonckheere et al., 2008
tRNA^Gly^	m.9997T>C	Nonobstructive cardiomyopathy	Oxygen consumption, complex I- and complex IV-specific activities, and lactate production, were markedly abnormal	590035	Merante et al., 1994
	m.10003T>C	Hypertension	Potential structural and functional alterations	590035	Xue et al., 2016
tRNA^His^	m.12192G>A	Cardiomyopathy	Morphological alteration of cardiac mitochondria and structural change	590040	Shin et al., 2000
tRNA^Glu^	m.14692A>G	Hypertension	Junction of T-stem and T-loop; Decrease in the steady-state level of tRNA^Glu^	590025	Xue et al., 2016
MT-CYB	m.14849T>C	Hypertrophic cardiomyopathy	Low alpha-tocopherol concentrations in his muscles and an elevated urinary leukotriene E(4) excretion indicate increased production of reactive oxygen species; amino acid change p.Ser35Pro in Cyb	516020	Schuelke et al., 2002
	m.15498G>A	Histiocytoid cardiomyopathy	Substitution of glycine with aspartic acid at amino acid position 251	516020	Andreu et al., 2000
MT-TT	m.15909A>G	Hypertension	D-stem of tRNA^Thr^; reduced mitochondrial protein synthesis; ATP decreased and the generation of ROS increased	590090	Xue et al., 2016

RETRACTED

### The Mitochondrial tRNA^Ile^ m.4263A>G and tRNA^Ala^ m.5655A>G Mutations Are Associated With EH

The tRNA^Ile^ m.4263A>G mutation (OMIM590045) has been reported in a Han Chinese family with EH (Wang et al., 2011). This mutation is located at the 5′ initiation site of tRNA^Ile^ (Figure 2), and thus may affect mitochondrial tRNA^Ile^ transcription and processing of the 5′ end by RNase P. Functional studies have shown that tRNA^Ile^ m.4263A>G mutations resulted in decreased mitochondrial oxygen consumption (Holzmann et al., 2008), and may contribute to the development of systematic hypertension (Marian, 2011). Similarly, tRNA^Ala^ m.5655A>G (OMIM560000) is located at the 5′ end of the tRNA precursors that is processed by RNase P, and its presence resulted in a 41% reduction in the steady-state level of tRNA^Ala^ in mutant cell lines (Jiang et al., 2016). Another study showed that the presence of this mutation results in a 29.1% reduction in the expression of six mtDNA-encoded protein that was associated with a significant decrease in ATP synthesis and mitochondrial membrane potential.

### The Mitochondrial tRNA^Met^ m.4435A>G Mutation Is Associated With EH

The mitochondrial tRNA^Met^ m.4435A>G (OMIM590065) mutation is located at position 37, adjacent to the anticodon, which is highly conserved (Sprinzl et al., 1998). This position is more easily modified than other sites, and plays a very important role in high fidelity anti-codon recognition, maintenance of tRNA tertiary structure, and biochemical function (Björk, 1995). Similarly, in *Escherichiacoli*, modification of the 37th position of tRNA^Lys^ plays a crucial role in stabilizing of the tRNA^Lys^ anti-codon (Li et al., 1997). Substitution of bases A with base G at position 37 can result in a significant reduction in tRNA aminoacylation (Yarus et al., 1986). The tRNA^Met^ m.4435 A>G mutation alter the tRNA^Met^ structure, conferring increased melting temperature and electrophoretic mobility and decreased aminoacylation efficiency and steady-state levels of tRNA^Met^ (Zhou et al., 2018). Further functional studies have found that the tRNA^Met^ m.4435A>G mutation results in an ~40% decrease in the amount of mature tRNA^Met^ that is expressed. This results in an ~30% reduction in mitochondrial protein translation. These studies also found that this decrease in transcription and translation affects the function of the mitochondrial respiratory chain, leading to reduced ATP synthesis and increases production of reactive oxygen species (ROS) (Liu et al., 2009).

### The Mitochondrial tRNA^Met^/tRNA^Gln^ m.4401A>G Mutation and EH

The mitochondrial tRNA^Met^/tRNA^Gln^ m.4401A>G (OMIM590065) mutation is located between the 5′ end of gene encoding tRNA^Met^ in the heavy strand and the gene encoding tRNA^Gln^ in the light strand (Ojala et al., 1981), which is a highly conserved in the evolution. Mitochondrial tRNAs are precisely cleaved at the 3′ and 5′ ends by RNase P and tRNase Z (Levinger et al., 2004; Holzmann et al., 2008; Wang et al., 2011), so this mutation may affect the processing efficiency of tRNA^Met^ and tRNA^Gln^. Further functional studies have found that the mitochondrial tRNA^Met^/tRNA^Gln^ m.4401A>G mutation causes an ~30% decrease in both tRNA^Met^ and tRNA^Gln^ expression, and an ~26% reduction in OXPHOS protein synthesis, as well as a decrease in NADH-ubiquinone oxidoreductase (complex I), ubiquinol-cytochrome c oxidoreductase (complex III), and cytochrome oxidase (complex IV) activity of ~78%, 78%, and 80%, respectively (Li et al., 2009).

RETRACTED

### Other Mutations Associated With EH

In 2004, Jones et al. reported that the tRNA^Leu(UUR)^ m.3243A>G (Jones et al., 2004) (OMIM590050) mutation is associated with hypertension, ischemic heart disease, and asthma. The mitochondrial ND1m.3308T>C mutation (Liu et al., 2008) (OMIM516000) replaces the start codon (methionine) with a codon encoding threonine, resulting in the production of a truncated MT-ND1 that is translated from a downstream methionine and lacks two amino acids. In addition, because MT-ND1 m.3308T>C is adjacent to the 3′ end of tRNA^Leu(UUR)^, it also affects the synthesis of tRNA^Leu(UUR)^ precursors (Li et al., 2004; Liu et al., 2008). The tRNA^Leu(UUR)^ m.3253T>C mutation (OMIM590050), identified in a Han Chinese family with EH, is located at position 22 in the D-stem, contributing to a G-C base pairing (G13-C22) at the D-stem and a tertiary base pairing (C22-G46) between the D-stem and the variable loop. This change is associated with a decrease in the steady-state level of tRNA^Leu(UUR)^ (Zhou et al., 2017). Linear mixed effects model analysis revealed that individuals from the FHS with the m.5913G>A (OMIM516030) mutations had a systolic BP that was an average of 7 mmHg higher at baseline than individuals without this mutation (*P*_empirical_ = 0.05) (Liu et al., 2012). To improve screening for mtDNA mutations that are associated with hypertension, we developed the following novel screening criteria: the mutation must (1) be present in <1% of controls; (2) be evolutionarily conserved; (3) have potential structural and functional effects. According to these criteria, tRNA^Gly^ m. 10003T>C (OMIM590035), tRNA^Asp^ m.7551A>G (OMIM590015), tRNA^Glu^ m.14692A>G (OMIM590025), and tRNA^Thr^ m.15909A>G (OMIM590090) are candidate variants associated with EH (Xue et al., 2016).

Cleavage of the 5′ end of mitochondrial tRNAs is related not only to the mitochondrial genome, but also to RNase P function. RNase P–mediated cleavage is affected by two main factors: mutations in mitochondrial tRNAs and mutation or abnormal expression of its protein subunits (MRPP1, MRPP2, and MRPP3). The protein subunits of RNase P are encoded by the TRMT10C, HSD17B10, and KIAA0391 nuclear genes, respectively. TRMT10C mutation affects tRNA^Phe^ and tRNA^Leu(UUR)^ steady-state levels, which, in turn, affects the expression of mitochondrial proteins involved in the respiratory chain, leading to defects in mitochondrial function. However, mutations in HSD17B10p have no effect on mitochondrial tRNA expression or function (Metodiev et al., 2016). K212E mutations affecting RNase P lead to aberrant cleavage of the 5′ end of the mitochondrial tRNA^Leu(UUR)^ and are associated with neurodegenerative diseases (Reinhard et al., 2015), whereas KIA0391 mutations affect RNase P function and result in abnormal post-translational modification of tRNAs. Abnormal expression of each RNase P subunit also affects its cleavage function (Reinhard et al., 2015).

RETRACTED

## Pathophysiology and Function of mtDNA Mutations in EH

For technical and other reasons, several key issues have not yet been clarified (Marian, 2011; Kirchner and Ignatova, 2015). Cardiomyocytes and smooth muscle cells are excitable cells that exhibit conductivity and contractility, and the mtDNA copy number, mutation frequency, and mitochondrial homeostasis of these cells are also significantly different compared with other cell types. Nuclear gene variations could affect mtDNA mutation phenotypes in patient lymphocytes. MtDNA mutation leads to increased oxidative stress and disruption of mitochondrial homeostasis, but the molecular mechanism by which these changes affect blood pressure and promote cardiac hypertrophy remains unclear.

### Mitochondrial Oxidative Stress and Hypertension

The mitochondria provide 95% of the energy needed for cell activities and play an especially important role in energy-consuming cells such as cardiomyocytes and neurons (Gunter et al., 2004). In addition, mitochondria are also involved in physiological activities such as apoptosis, cell cycle regulation, and cell development. Mitochondria-mediated cell death (apoptosis) regulates ROS production and cell signal transmission, as well as intracellular calcium homeostasis (McFarland et al., 2007). Therefore, mitochondrial injury and dysfunction can have substantial effects on overall cell function. An increasing body of evidence suggests that hypertensive myocardial injury is closely related to abnormal mitochondrial function, mitochondrial structure, energy metabolism, and homeostasis in cardiomyocytes (Eirin et al., 2014; Gong et al., 2014). In a renin-induced rat model of hypertension and impaired cardiac function, mitochondrial degeneration and swelling were accompanied by changes in mitochondrial density and structure (Walther et al., 2007). In addition, the activity of cardiomyocyte complex coenzyme III, ATP synthase, and creatine kinase was decreased. Furthermore, cytochrome C release was increased, and caspase-3 expression was up-regulated, leading to increased apoptosis. Previously, Gong et al. (2014) found that tRNA mutations in patients with deafness could destabilize the secondary clover structure of tRNAs, leading to identification and transport of incorrect amino acids and ultimately disrupting mitochondrial OXPHOS peptide synthesis.

RETRACTED

ROS is a major factor contributing to oxidative stress in the body. As an important intracellular and intercellular regulatory factor, ROS plays a key role in the pathogenesis of hypertension and can lead to proliferation and migration of vascular smooth muscle cells (VSMC) and overexpression of inflammatory mediators and extracellular matrix. In addition, an increase in ROS leads to an increase in free calcium in endothelial cells, leading to vasodilatory dysfunction. Angiotensin II (AngII) can promote ROS synthesis by cardiomyocyte mitochondria, resulting in loss of mtDNA and increased autophagy (Dai et al., 2011b) In a mouse model of catalase overexpression, an antioxidant polypeptide that specifically targets the mitochondria (SS-31) can reduce myocardial damage, inhibit cardiac hypertrophy and fibrosis, and reverse the mitochondrial damage caused by Ang-II. In a stress-induced hypertensive rat model, the increase in mitochondrial ROS production by left ventricular cardiomyocytes leads to myocardial cell dysfunction and myocardial fibrosis (Dai et al., 2011a).

ROS, which are typically present in cells at low concentrations, are important signaling molecules that maintain vascular integrity by regulating endothelial function and vascular contraction–relaxation (Touyz et al., 2003). Under pathological conditions, ROS levels increase significantly, and can damage hypertensive vascular endothelial cells (Taniyama and Griendling, 2003). The tRNA^Ile^ m.4263A>G mutation contributes to disorders of respiratory complexes I, III, and IV, which are significantly enriched in AUC and/or AUU codons that pair with tRNA^Ile(GAU)^, thereby reducing substrate-dependent oxygen consumption to 70%−80% of normal levels (Kirchner and Ignatova, 2015). Increased ROS levels can damage the mitochondrial respiratory chain and mtDNA, leading to further mitochondrial dysfunction and cell death (Figure 3). Several animal studies have shown that high BP is alleviated by inhibiting mitochondrial ROS generation, providing clear evidence of the association between hypertension and oxidative stress (Liang, 2011). Moreover, a recent study found that cybrids harboring the m.1494C>T mutation contain more dysfunctional mitochondria than wild-type cells, resulting in mitochondrial fusion and mitophagy (Yu et al., 2014), which may contribute to cardiomyocyte apoptosis and ventricular and vessel remodel (Figure 3).

RETRACTED

**Figure 3:** Potential mechanisms involved in tRNA mutation-associated EH, altered ROS synthesis, and ATP synthesis defects. MtDNA mutation leads to decreased tRNA expression, inhibition of mitochondrial OXPHOS-related protein synthesis, increased mitochondrial oxidative stress, increased cell apoptosis, leading to vascular remodeling. Dysfunctions of OXPHOS in mitochondria lead to abnormal energy metabolism and abnormal changes in the exchange of sodium and calcium, leading to calcium overload in the cytoplasm, diastolic dysfunction of cardiomyocytes and smooth muscle cells, and promoting blood pressure increase.

### Mitochondrial Energy Synthesis Disorders and Hypertension

Postnov et al. observed that the rate of ATP synthesis was significantly lower in rats with spontaneous hypertension than in control animals (Doroshchuk et al., 2004). Disorders of complexes I, III, or IV that disrupt respiration decrease the mitochondrial proton electrochemical potential gradient and inhibit mitochondrial ATP synthesis (Figure 3). Large mtDNA deletions or tRNA mutations disrupt the respiratory chain and decrease the proton electrochemical potential gradient as well as the capacity for ATP synthesis. A recent study showed that ATP production in mutant cell lines carrying the tRNA^Leu(UUR)^ m.3253T>C mutation was 66% lower than the mean control value (Zhou et al., 2017). Oxidative phosphorylation defects that completely block mitochondrial ATP synthesis are fatal, as shown by knocking out transcription factor A expression in mice (Larsson et al., 1998), which may be associated with disturbance of excitatory contraction coupling in cardiomyocytes and smooth muscles.

### Mitochondrial Calcium Cycle Regulation Disorder and Hypertension

Despite considerable effort, including recent molecular and genetic biology studies, the exact molecular mechanism underlying hypertension is poorly understood. Postnov (Postnov et al., 1980) observed a significant increase in exchangeable intracellular calcium in adipose tissue from patients with EH. Cytosolic Ca^2+^ can be affected by mitochondria either directly or indirectly. The direct path involves Ca^2+^ uptake into mitochondria via a mitochondrial calcium uniporter (MCU). Chen et al. observed that lower expression of MCU in cells with the tRNA^Ile^ m.4263A>G mutation contributed to dysregulated Ca^2+^ uptake into the mitochondria, and thus cytoplasmic Ca^2+^ overload (Chen et al., 2016). Similarly, (Boczonadi et al., 2018) reported that mutation of nuclear-encoded glycyl-tRNA synthetase gene (GARS) affects mitochondrial calcium metabolism and ER–mitochondria interactions which contribute to the neuron-specific clinical presentations. The indirect path involves ATP-dependent Ca^2+^ transport out of the cell or into intracellular stores (Figure 4). Therefore, both a decrease in ATP synthesis caused by mtDNA mutations and collapse of the mitochondrial membrane potential could lead to excessive cytosolic Ca^2+^ or calcium dyshomeostasis. Ca^2+^ overload may also lead to systolic/diastolic dysfunction in smooth muscle and apoptosis (Figure 3) (Duchen, 2000).

RETRACTED

**Figure 4:** MCU involved in mitochondrial calcium cycle disorder. Mitochondrial dysfunction leads to decreased ATP synthesis and increased ROS, leading to intracellular calcium overload and altered MCU activity. Intracellular calcium overload leads to dysregulation of excitation–contraction coupling of vascular smooth muscle cells, which inhibits vasodilation and leads to hypertension.

In a hepatic ischemia-reperfusion injury (IRI) in rats, ROS initiates MCU opening, leading to increased apoptosis. Vecellio found that MCU plays an important role in the transport of calcium ions between the mitochondria and the sarcoplasmic reticulum in skeletal muscle cells (Vecellio et al., 2016). Knock-out of BNIP3, which encodes a protein related to myocardial cell mitochondrial autophagy, showed that BNIP3 regulates the mitochondrial calcium cycle in rats by affecting mitochondrial outer membrane channel protein expression (Chaanine et al., 2013), which leads to Ca^2+^ transport in the endoplasmic reticulum (ER), mitochondrial injury, increased apoptosis, and left ventricular myocardial fibrosis. A recent study further confirmed that MCU inhibitors can inhibit mitochondrial autophagy in neurons in the ischemia/reperfusion model, proving that MCU plays an important role in regulating mitochondrial autophagy (Yu et al., 2016). This mechanism may partially explain the pathogenesis of hypertension associated with mtDNA mutations.

## Conclusions and Prospects

Several hypertension-related tRNA mutations have been reported, including tRNA^Leu(UUR)^ m.3243A>G and m.3253T>C; tRNA^Met^/tRNA^Gln^ m.4401A>G; tRNA^Ile^ m.4291T>C, m.4295A>G, and m.4263A>G; tRNA^Met^ m.4435A>G; tRNA^Ala^ m.5655 A>G; tRNA^Asp^ m.7551A>G; tRNA^Gly^ m.10003T>C; tRNA^Glu^ m.14692A>G; and tRNA^Thr^ m.15909A>G. These mutations affect tRNA transcriptional modification and translation, and thereby contribute to the occurrence and development of hypertension. The identification of the mutation site is helpful for the diagnosis and early treatment of maternal hereditary hypertension, thus reducing the damage of target organs in the next generation of hypertension. While some hypotheses have been suggested to explain the molecular mechanism underlying mtDNA mutation-associated EH, they have yet to be definitively proven. EH is a disease with complex pathology that involves maternal inheritance, nuclear interactions, and environmental factors. Exploration of the underlying molecular mechanism has been hampered by the difficulties of generating an animal model of mitochondrial genetic disease containing accurate gene knock-outs or induced mutations. Recent developments in the use of induced pluripotent stem cells (iPSCs) and human umbilical vein endothelial cells (HUVECs) have promising implications for the study of mtDNA mutation-related diseases. We predict that the development of advanced molecular biochemical methods, including iPSCs and mitochondrial fusion cell lines constructed using HUVECs, will enable the detailed mechanisms of mtDNA-related EH to be elucidated in the future.

RETRACTED

## Author Contributions

All authors listed have made a substantial, direct and intellectual contribution to the work, and approved it for publication.

## Conflict of Interest

The authors declare that the research was conducted in the absence of any commercial or financial relationships that could be construed as a potential conflict of interest.
